# Influence of P(VDF-TrFE) Membranes with Different Surface Potentials on the Activity and Angiogenic Function of Human Umbilical Vein Endothelial Cells

This article has been retracted.

**DOI:** 10.1155/2022/5693994

**Published:** 2022-09-26

**Authors:** Yan Xu, Mingwei Cheng, Peijun Zhu, Shuo Yang, Chunhua Lai, Shulan Xu

**Affiliations:** Stomatology Hospital, Southern Medical University, Guangzhou 510280, China

## Abstract

During bone tissue regeneration, neovascularization is critical, and the formation of a blood supply network is crucial for bone growth stimulation and remodeling. Previous studies suggest that bioelectric signals facilitate the process of angiogenesis. Owing to their biomimetic electroactivity, piezoelectric membranes have garnered substantial interest in the field of guided bone regeneration. Nevertheless, the knowledge of their influence due to varying surface potentials on the progression of angiogenesis remains ambiguous. Therefore, we proposed the preparation of an electroactive material, P(VDF-TrFE), and investigated its effects on the activity and angiogenic functions of human umbilical vein endothelial cells (HUVECs). The HUVECs were directly cultured on P(VDF-TrFE) membranes with different surface potentials. Subsequently, cell viability, proliferation, migration, tube formation, and expressions of related factors were assessed through appropriate assays. Our results revealed that the negative surface potential groups exerted differential effects on the modulation of angiogenesis *in vitro*. The P(VDF-TrFE) membranes with negative surface potential exhibited the greatest effect on cellular behaviors, including proliferation, migration, tube formation, and promotion of angiogenesis by releasing key factors such as VEGF-A and CD31. Overall, these results indicated that the surface potential of piezoelectric P(VDF-TrFE) membranes could exert differential effects on angiogenesis *in vitro*. We present a novel approach for designing bioactive materials for guided bone regeneration.

## 1. Introduction

Guided bone regeneration (GBR), a standard therapeutic procedure, combines bone augmentation with a barrier membrane for the repair of maxillofacial bone defects [1]. The GBR barrier membrane preserves the spatial integrity of the graft filler and inhibits the invasion of the gingival fibrous tissues in the bone healing region, thus facilitating bone regeneration. Thus far, bioinert GBR barrier membranes have been utilized in several contexts in clinical settings, including the treatment of alveolar bone defects caused due to periodontitis, malignancies, and maxillofacial trauma [2, 3]. Owing to the biological processes underlying GBR therapy and the novel concept of bioactive materials, bioactive barrier membranes can stimulate the formation and regeneration of new bone.

Angiogenesis is a key component in bone growth and remodeling [4]. In addition to delivering nutrients, growth factors, hormones, cytokines, and chemokines to bone tissues and eliminating waste products, the bone vasculature also serves as a communication network between the bone and nearby tissues [5, 6]. Given the close spatial and temporal association between bone formation and vascularization, a barrier membrane with proangiogenic activity is a promising strategy for improving bone regeneration and repair.

Endogenous electrical signals promote tissue regeneration and reconstruction (C. [7, 8]; Z. [9, 10]). Previous studies show that external electrical stimulation modulates or promotes angiogenesis through relevant cellular behaviors (M. [11]; H. [12]). Furthermore, the application of electroactive biomaterials as mediators of electrical signals to promote angiogenesis has been reported previously ([13]; W. [14]). The application of this method in clinical settings is restricted due to its inefficiency and discomfort. Inherently, electroactive biomaterial implantation is a potential technique for localized electrical stimulation to address the above problem. Piezoelectric materials are smart materials that can produce electrical activity due to deformations or an external electric field [15]. This characteristic allows the delivery of electrical stimuli without external power. These piezoelectric polymers have been tested *in vitro* and *in vivo* for tissue regeneration owing to their biomimetic electroactivity ([16]; Y. [17]).

Previous studies have focused on the cytotoxicity and biocompatibility of piezoelectric polymers [18, 19]. However, studies on cell-biomaterial interactions are essential for the evaluation of their utility. Cellular phenomena related to biomaterials include cell adhesion, spreading, and proliferation [20]. Cell adhesion to the matrix is the initial and key process in tissue engineering as it affects subsequent cell behaviors and viability [21]. The adhesion of cells to the surface of biomaterials is the main factor regulating their biocompatibility. The surface properties of biomaterials can guide complex processes underlying cell adhesion, and the functionalization of the surface can control both cell morphology and responses [22]. Initial cell adhesion, determined by electrostatic forces, is crucial for cell communication and tissue development. The surface charge and potential determine the number, type, and degree of refolding of absorbed proteins and the subsequent cell adhesion processes [23]. Accumulating evidence on cell-matrix interfaces and the rapid development of tissue engineering has prompted our study on the surface potential in detail for different types of biological materials (W. [24]). Each cell type has unique properties, including the actual cellular responses to surface charge [25]. Such specific properties allow the designing and adaptation of biomaterial surfaces for specific applications. However, the influence of piezoelectric materials on cellular angiogenesis remains largely unclear. Moreover, to improve the development of piezoelectric GBR membranes, it is critical to determine whether their differential surface potential characteristics affect cell behavior.

This work aimed to contribute to our understanding of the effects of different surface potentials on the cellular behavior and angiogenesis processes of human umbilical vein endothelial cells (HUVECs) *in vitro*. Owing to its high electrical activity, physicochemical properties, and good biocompatibility, the P(VDF-TrFE) membrane was chosen as the experimental material in this study. Furthermore, P(VDF-TrFE) membranes with different surface potentials were synthesized, and their effects on the function of HUVECs were assessed.

## 2. Materials and Methods

### 2.1. Fabrication and Characterization of P(VDF-TrFE) Membranes

The P(VDF-TrFE) membranes were synthesized as described previously [26]. Briefly, 3 grams of powdered P(VDF-TrFE) polymer (Arkema, Paris, France) was dissolved in 20 milliliters of N,N-dimethylformamide (Aladdin, Shanghai, China) and dissolved at 60 °C. Subsequently, the solution was deposited on a titanium substrate and dried at 80 °C to allow the evaporation of the solvent, followed by isothermal crystallization. The P(VDF-TrFE) membranes were poled with a direct current electric field (6 kV/cm, 60 min, at 120 °C). The samples were divided into three groups based on their surface potential, “nonpoled”, “ negative (poled -)”, and “ positive (poled +).”

Scanning electron microscopy (SEM; Gemini 300, Zeiss, Germany) was performed to observe the surface morphology. The water contact angles of the samples were tested using a contact angle goniometer (ZhongChen Co., Ltd, Shanghai, China). X-ray diffraction (XRD, Ultima VI, Shimadzu, Kyoto, Japan) and Fourier transform infrared spectroscopy (FTIR, Bruker Optik GmbH, Ettlingen, Germany) analyses were also performed to determine the influence of polarization on the crystal structures. Subsequently, the relative surface potential of the poled P(VDF-TrFE) membranes was assessed by Kelvin probe force microscopy (KPFM, AFM, Brucker Icon, Billerica, USA). The P(VDF-TrFE) membrane without polarization (“nonpoled”) was the control group.

### 2.2. Cellular Responses to P(VDF-TrFE) Membranes with Differential Surface Potentials

#### 2.2.1. Cell Culture

HUVECs were cultured in Dulbecco's modified eagle medium (DMEM) with high glucose (Thermo Fisher Scientific, USA) supplemented with 10% fetal bovine serum (FBS, ExCell Bio Company, Shanghai, China) and 1% penicillin-streptomycin solution (Thermo Fisher Scientific, USA) under standard growth conditions (5% CO_2_, 37 °C, and humidified sterile environment). Cells were then digested with trypsin-EDTA (0.25%) (Thermo Fisher Scientific, USA) for subsequent steps.

#### 2.2.2. The Direct Contact Test

The samples were sterilized by immersing in 75% ethanol overnight and exposed to UV light for 1 h before the experiment. The direct contact test was evaluated through two biological assays for cell membrane integrity and morphology (KGAF001, KeyGEN BioTECH, China) and cell proliferation (CCK-8, Dojindo, Japan). Cells without samples were used as the control. The cells were seeded onto a 24-well plate at a density of 1.25 × 10^4^ cells/cm_2_. After 24 h of incubation, the wells were rinsed twice in phosphate buffer solution (PBS, Thermo Fisher Scientific, USA). The cells were incubated in dark for 30 minutes with a 1 mL working solution (containing 4 *μ*M calcein and 8 *μ*M propidium iodide in 10 mL of PBS). The samples were then examined under a fluorescence microscope (Optiphot-2, Nikon Corporation, Tokyo, Japan). For the determination of proliferative ability, cells were seeded in the samples at a density of 5 × 10^4^ cells/cm_2_. After incubation for 24 h and 72 h, the medium was replaced with a medium containing 10% CCK-8 solution and incubated for another 2 h. Next, 100 *μ*L of the medium per well was transferred to a 96-well plate. The absorbance was measured at 450 nm using a microplate reader (ELX808, Bio-Tek, USA).

#### 2.2.3. Cell Migration

The cell scratch and wound healing assay was performed to evaluate the effect of differential surface potentials on cell migration. The cells were seeded onto different samples in a 6-well plate at a density of 1 × 10^4^ cells/cm_2_. The scratch was made using a sterile pipette tip when the cell confluency reached 90%. The scratch width of every group was kept consistent at nearly 2 mm. After incubation for 6 h, 12 h, and 24 h, cells were examined under an optical microscope (DM4000, Leica, German). Images were quantitatively assessed using ImageJ 1.51.

#### 2.2.4. Tube Formation Assay

The tube formation assay was performed to determine the effect of surface potentials on the angiogenesis of HUVECs *in vitro*. The sterilized pipette tips were pre-chilled to − 20 °C, and the Matrix gel (BD Biosciences, Bedford, MA, USA) was thawed overnight at 4 °C. After preparation, the liquefied matrix gel was carefully aspirated using the pre-chilled tips and evenly coated on the 48-well plate; care was exercised to not let in air bubbles. All steps were carried out on the ice to prevent the solidification of the Matrix gel at high temperatures. To guarantee consistency in Matrix gelation, the 48-well plates were placed in an incubator at 37 °C with 5% CO_2_ for 30 minutes. HUVECs following different treatments during co-culture were digested, centrifuged, and resuspended in 1 ml of the medium while waiting for the matrix gel to harden. Subsequently, 1 mL of the cell suspension was added to each well of the 48-well plate with solidified matrix at a density of 1 × 10^5^cells/cm^2^ (making sure to thoroughly mix the addition by blowing with a pistol tip before adding). After the procedure, the 48-well plate was incubated at 37 °C with 5% CO_2_ for 4–6 h to detect tube development in HUVECs. The tubes were observed under a microscope.

#### 2.2.5. Effects of P(VDF-TrFE) Membranes with Differential Surface Potentials on Gene Expression

After 48 h of co-culture with the samples, total RNA was isolated from HUVECs using AG RNAex Pro reagent (AG21101, Accurate Biotechnology, Hunan, China). The amount and purity of the RNA were measured on a Nanodrop 100 spectrophotometer. The Evo M-MLV RT Kit with gDNA Clean was utilized to remove genomic DNA for qRT-PCR. Subsequently, reverse transcription was conducted. The SYBR Green Premix Pro Taq HS qPCR Kit (AG11701, Accurate Biotechnology, Hunan, China) was used to perform qRT-PCR following the manufacturer's protocol. The expressions of genes of interest, including vascular endothelial growth factor A (VEGF-A) and platelet endothelial cell adhesion molecule-1 (CD31), were quantified. Glyceraldehyde-3-phosphate dehydrogenase (GAPDH) was used as a normalization control. The primer sequences used in the study are listed in Table 1.

#### 2.2.6. Effects of P(VDF-TrFE) Membranes with Differential Surface Potentials on Protein Expression

In 6-well plates, cells were co-cultured with the samples for 48 h. Total proteins were extracted from the cells using a RIPA lysis buffer (P0013, Beyotime Biotechnology, China). According to standard protocols, protein extracts were resolved by 8% SDS-PAGE and transferred onto PVDF membranes (Bio-Rad, Hercules, USA). PVDF membranes were blocked for 1 h with BSA containing 5% non-fat dry milk. Subsequently, PVDF membranes were incubated overnight at 4 °C with primary antibodies (GAPDH (1 : 1,000, Boster, China), VEGF-A (1 : 1,000, Proteintech, China), and CD31 (1 : 1,000, Proteintech, China)) followed by incubation with secondary anti-rabbit or anti-mouse IgG (1: 2000) for 1 h after washing them twice in TBST. The membranes were treated with an enhanced chemiluminescent agent to detect the protein bands (ECL, Pierce, USA). The Image Lab 4.1 software was used to analyze the data (Bio-Rad Laboratories, Hercules, CA, USA).

### 2.3. Statistical Analysis

Biological results were determined following three independent experiments. All data sets were analyzed using the GraphPad PRISM Version 9.00 software (GraphPad Software, Inc., USA). Considering the different polarization procedures and time as independent factors, a two-way analysis of variance (ANOVA) was used to evaluate the numerical data, followed by Tukey's multiple comparison post hoc test for differential polarization treatments at the same time point. Wherever applicable, one-way ANOVA was used to analyze data from three or more groups, followed by Dunnett's multiple comparison post hoc test. Statistical significance was defined at *P* value < 0.05.

## 3. Results

### 3.1. Characterization of P(VDF-TrFE) Membranes

A direct current field was used to pole the P (VDF-TrFE) membranes used in this study, following which FTIR and XRD analyses were performed to determine the *β*-phase content in the materials. Compared to the nonpoled group, both poled groups exhibited typical *β*-phase FTIR peaks (840 cm^−1^ and 1400 cm^−1^) (Figure 1(a)). XRD analysis (Figure 1(b)) showed that the poled groups exhibited a prominent peak at approximately 20° relative to the nonpoled group, indicating an abundance of *β*-phase content. Overall, the content of the *β*-phase increased following negative and positive polarization.

As shown in Figure 2(a), SEM images reveal that the surface of P(VDF-TrFE) membranes was smooth, with no obvious fractures or defects, suggesting that polarization did not change or damage the surface morphology; no significant differences in the surface morphology among the groups was observed. The surface water contact angles (Figure 2(b)) of the P(VDF-TrFE) membranes after polarization were less than 90°, and no significant differences were found among groups, demonstrating that polarization did not change the wettability of the material surface.

The surface potentials of P(VDF-TrFE) membranes were characterized by AFM. As shown in Figure 3, the surface potential of the negative group is −2.11 ± 0.10 V; it is +2.59 ± 0.90 V for the positive group and −0.551 ± 0.245 V for the nonpoled group. These results indicated that the surface potentials of the P(VDF-TrFE) membranes changed after polarization. The differentially poled groups developed different surface potentials.

### 3.2. HUVECs in the Direct Contact with P(VDF-TrFE) Membrane

As shown in Figure 4(a), live-dead assay was performed to assess the influence of direct contact of HUVECs with the differentially poled P(VDF-TrFE) membranes. After 24 h of direct contact incubation, fluorescence images of HUVECs co-cultured in different groups were analyzed (Figure 4(a)). Most cells showed spindle-shaped morphology (green fluorescence), and only a few dead cells (red fluorescence) were observed in all poled groups. Cells in the nonpoled group showed a good-shaped morphology with no significant differences from those in the control group. Therefore, P(VDF-TrFE) membranes with differential surface potentials did not negatively affect the viability of HUVECs.

The CCK-8 assay was performed to further elucidate the effects of differentially poled P(VDF-TrFE) membranes on cell proliferation (F (3, 48) = 3.107, *p* = 0.0350).  Figure 4(b) illustrates the relative proliferation of cells incubated for 24 and 72 h. The results showed that after 24 h, the negative group and the control group exhibited similar proliferation levels with no statistically significant differences. At 72 h, the negative group showed the highest level of proliferation as compared to the other groups, and the difference was statistically significant (nonpoled: *p* < 0.0001; control: *p* < 0.0001).

### 3.3. Effects of P(VDF-TrFE) Membranes with Differential Surface Potentials on Cell Migration

The results of the P(VDF-TrFE) membranes with differential surface potentials on cell migration are summarized in Figure 5. A two-way ANOVA test suggested that the effects of differentially poled P(VDF-TrFE) membrane over time on cell migration were significant (F (9, 36) = 7.438, *p* < 0.0001). As shown in Figure 5(a), the initial scratch width in all groups was consistent at nearly 2 mm. After 6 h, the scratch area decreased slightly in all groups. No statistically significant differences were observed at this time point. Relative to the control group, the wound area left unhealed in the poled groups (*p* = 0.0005) and nonpoled groups (*p* = 0.0271) at the 12 h time point also decreased significantly. At 24 h, the negative group and nonpoled group showed a significant reduction in the wound area left unhealed as compared to the control group (poled - groups: *p* = 0.0003; nonpoled group: *p* = 0.0180). Wound closure was not 100% at the end of 24 h. Wound closure in the control, nonpoled, positive, and negative groups were 52.19 ± 3.629%, 69.76 ± 6.211%, 67.27 ± 7.181%, and 85.90 ± 1.331%, respectively. Taken together, these results suggested that the membrane with negative surface potential significantly enhanced the migration of HUVECs.

### 3.4. Effects of P(VDF-TrFE) Membranes with Differential Surface Potentials on Tube Formation

Tube formation is critical in angiogenic processes. The possible impacts of varying surface potentials on HUVEC tube formation *in vitro* were investigated by a tube formation assay (Figure 6). After incubation for 6 h, sturdy and elongated tube-like structures developed when HUVECs were incubated in Matrigel pre-coated 48-well plates. The length of the main stem of the formed tubules was quantified using the Image J software (F = 7.024, *p* = 0.0125). Unsurprisingly, negative group promoted tube formation, whereby the length of the main segment was significantly greater than those in the control and positive groups (poled +: *p* = 0.0059; control: *p* = 0.0311). These results demonstrated the potential of the membrane with negative surface potential to promote tube formation *in vitro.*

### 3.5. Effects of P(VDF-TrFE) Membranes with Differential Surface Potentials on Angiogenesis-Related Factor Expression

In this study, the expressions of the angiogenesis factors, VEGF-A and CD31, were analyzed by qRT-PCR (Figure 7) and western blotting. The statistical differences among the groups were confirmed using one-way ANOVA (VEGF-A: F (3, 32) = 5.473, *p* = 0.0038; CD31: F (3, 44) = 4.732, *p* = 0.0060). Dunnett's multiple comparisons test revealed that the negative group showed the highest level of VEGF-A expression as compared to the positive group (*p* = 0.0081), nonpoled group (*p* = 0.0125), and control group (*p* = 0.0032). The gene expression of CD31 exhibited similar trends. The gene expression of CD31 in the negative group was significantly higher relative to those in the others (poled + group: *p* = 0.0248; nonpoled group: *p* = 0.0057; control group: *p* = 0.0090). To further confirm the effects of differential surface potential membranes on angiogenesis, the levels of protein expression of CD31 and VEGF-A were determined by western blotting (Figure 8). According to quantitative data analysis, the trend of VEGF-A protein expression was consistent with those of the corresponding mRNA levels. The level of VEGF-A expression in the negative group increased significantly (control: *p* = 0.0395; poled +: *p* = 0.0251; nonpoled: *p* = 0.0075), which implied that the membrane with negative surface potential promoted the secretion of VEGF-A.

## 4. Discussion

In this study, piezoelectric P(VDF-TrFE) was poled by direct current fields, thereby generating differential surface potentials in these materials. The FTIR and XRD results showed that the *β*-phase content increased, consistent with the findings of a previous study. Cell behavior can be influenced by the surface morphology and wettability of biomaterials [20]. Previous studies suggest that the surface contact angle and surface topography affect the cell's attachment and proliferative abilities [27, 28]. However, based on our results, no significant differences in surface contact angle and topography of P(VDF-TrFE) films before and after polarization were observed. Therefore, the findings exclude the effects of the topography and wettability of biomaterials on cell behavior.

Biocompatibility is the ability of a biomaterial to elicit an adequate host response, crucial for its clinical applicability. Electroactive biomaterials are promising bioactive materials; thus, they have gained increasing interest owing to their biological safety. Several studies suggest that biocompatible piezoelectric materials can serve as tissue stimulators and scaffolds to promote tissue regeneration [19, 29]. As a non-biodegradable biomaterial, good biocompatibility is crucial to achieving long-term retention in the body for widespread utility. Therefore, the biosafety of electroactive P(VDF-TrFE) membranes must be carefully evaluated and considered. Moreover, the dynamic interaction between endothelial cells and material is complex, and the surface properties of biomaterials critically influence this dynamic interaction. The surface potential of biomaterials is an important regulatory factor for cellular responses and cell signaling in tissue therapy [20]. For a biomaterial with good piezoelectric and ferroelectric properties, the surface potential developed after polarization also affects the behavior of HUVECs. We analyzed the effects of electroactive P(VDF-TrFE) membranes on the cell viability of HUVECs by a dead-live assay. No significant cytotoxicity or effects on cell viability in HUVECs were observed for the P(VDF-TrFE) membranes. The good performance of P(VDF-TrFE) membranes as biomaterials was also preliminarily confirmed. This result is consistent with those reported previously by Hitscherich [16].

To better understand the effects of P(VDF-TrFE) membranes with different surface potentials on the proliferation of HUVECs, the CCK-8 assay was performed for quantification. All groups showed good biocompatibility. In particular, the negative groups significantly promoted the proliferation of HUVECs relative to the control group. Similar trends have been reported by Szewczyk for PVDF fibers with different surface potentials. The scaffolds built using PVDF (-) fibers show greater potential for bone regeneration than PVDF (+) [30].

In addition to cell proliferation, endothelial cell migration is also important for angiogenesis [31]. Upon blood vessel injury, endothelial cells migrate to fill the resulting open space and restore the structural integrity of the vessels [32]. Thus, a cell proliferation assay provides the most direct and interpretable data. However, these only represent a part of events during angiogenesis and do not capture the entire process. The formation of new blood vessels can occur through rapid cell multiplication and is triggered by cell migration. Thus, cell migration was evaluated. The scratch–wound assay was performed to evaluate the effects of different surface potentials on cell migration. Notably, the negative group was the most effective in increasing cell migration relative to the other membranes. This general trend is in line with the results obtained for cell proliferation. Interestingly, previous studies suggest that electrical stimulation guides endothelial cell migration toward the anode (M. [11]; M. [33]). Similarly, electrical stimulation benefits the proliferation of HUVECs on a conductive scaffold [13]. The impact is related to the voltage output of the biomaterials.

During angiogenesis, VEGF-A plays an equally active role as a growth factor with important pro-angiogenic effects. It triggers the proliferation and migration of endothelial cells, induces tubulogenesis, promotes endothelial cell survival, and inhibits apoptosis ([34]; X. [35, 36]). Previous studies report that endogenous electrical stimulation affects VEGF release from HUVECs *in vitro*, thereby increasing the mRNA expression of VEGF (H. [12]). In the present study, the level of VEGF-A expression was examined and was found to be significantly upregulated in the negative group, consistent with the results of previous experiments indicating that the negative group promoted cell proliferation, migration, and tube formation in HUVECs, possibly by regulating the expression of VEGF-A. Zhao et al. (Q. [37]) also prepared scaffolds with different surface potentials by the electrostatic spinning of emulsions using power supplies with different polarities. Scaffolds made with negative voltage emulsions better promoted endothelial cell functions, consistent with our results. In the present study, we analyzed the level of CD31 expression, an important angiogenic marker by qRT-PCR and western blotting. The gene expression of CD31 was significantly upregulated in the negative group relative to other groups. Protein expression of CD31 was also upregulated in the negatively poled group. This suggests that the P(VDF-TrFE) membranes with negative surface potential are likely to affect the level of CD31 expression, thus influencing the migration of HUVECs and the formation of tubular structures *in vitro*.

The surface of the poled P(VDF-TrFE) electroactive membrane generated differential surface potentials. According to the ion attraction in the electric double layer, when different groupings of samples are immersed in the medium simulating the *in vivo* environment, some ions are selectively adsorbed onto the sample surface owing to electrostatic reactions [38]. Specifically, on the surface of samples with negative surface potential, cations and positively poled ionic groups are actively adsorbed (W. [39]). The VEGF-A protein exhibits positive electrical properties, and thus, it adhered to the surface of the negative group owing to the electrostatic interaction. The deposition of calcium ions on negative surfaces further formed a cationic layer, consequently promoting the adhesion of proteins and cells [40]. The surface of the nonpoled group was electrically neutral and did not attract inorganic ions, amino acids, proteins, and other substances floating in the medium and, thus, did not affect the adhesion and function of cells or proteins relative to the polarized samples.

Previous studies suggest that the electrical properties of piezoelectric materials contribute to the formation of cellular actin bundles and maturation of adherent spots, which further positively regulates cellular maturation and cellular piezoelectric self-stimulation and induces intracellular calcium transients [41]. Increased calcium ion concentration has long been recognized as a key pro-angiogenic mechanism underlying the intersection of multiple signaling cascades and is recruited by different mitogens to promote and regulate endothelial cell fate. Moreover, growth factors and chemokines induce an angiogenic switch by increasing the calcium ion concentration to stimulate endothelial cell proliferation, adhesion, migration, and tube formation [42]. This may partially explain why biomaterials with different surface potentials exert differential effects on the behavior of HUVECs. However, this is only a speculative hypothesis based on our results, and more experiments are needed to verify it. Future experiments to elucidate the mechanism of action are necessitated to better understand the principle of action underlying piezoelectric materials.

In this study, biomaterials with differential surface potentials were found to affect cell behavior and angiogenesis *in vitro*. Based on our analysis of the P(VDF-TrFE) membranes with differential surface potentials over months without any additional biochemical modifications, the P(VDF-TrFE) membranes with differential surface potentials were found to promote angiogenesis for tissue regeneration, a research hotspot in the field of bone regenerative medicine. However, the exact underlying mechanism remains unclear, and although an increasing trend of expression of some important markers was detected, further experiments are needed to investigate the mode of action to better understand this biomaterial for promoting its future application in the clinical settings.

## 5. Conclusion

In conclusion, differentially poled P(VDF-TrFE) membranes were prepared and characterized for the effects of electrical surface potentials of piezoelectric P(VDF-TrFE) on cellular behaviors and angiogenesis in HUVECs. Differentially poled P(VDF-TrFE) membranes triggered different cell behaviors in HUVECs. In summary, piezoelectric materials with differential surface potentials showed significant differences in regulating the functional secretion from HUVECs, which in turn affected subsequent angiogenesis processes. P(VDF-TrFE) membranes with negative surface potential showed better enhancement of angiogenesis. These findings have important implications for piezoelectric materials as a promising technique for guided bone regeneration with proangiogenic activity.

## Figures and Tables

**Figure 1:** Piezoelectric characterization of P(VDF-TrFE) membranes. (a), (b) The FTIR spectra and XRD patterns for P(VDF-TrFE) membranes before and after polarization, showing the amount of electroactive *β*-phase.

**Figure 2:** SEM images and Water contact angle of P(VDF-TrFE) membranes. (a), (b) SEM images and water contact angle for P(VDF-TrFE) membranes before and after polarization.

**Figure 3:** Physical characterization of differently poled P(VDF-TrFE) membrane. The KPFM images depict the distribution of relative surface potential for positively, negatively, and neutrally P(VDF-TrFE).

**Figure 4:** Effect of P(VDF-TrFE) membranes with differential surface potentials on cell morphology and proliferation. (a) The fluorescent representative images were observed after HUVECs in direct contact with the P(VDF-TrFE) membranes with differential surface potentials for 24 h, stained by AM/PI. The red fluorescence depicts apoptotic cells stained by PI, while the green fluorescence shows live cells with membrane integrity identified by AM (scale bar = 200 *μ*m). (b) Quantitatively cell viability was measured by CCK-8 assay. A two-way ANOVA is used to analyze the data that come from three independent tests. ^∗∗∗∗^*p* < 0.0001.

**Figure 5:** Effects of P(VDF-TrFE) membranes with differential surface potentials on cell migration by scratch wound assay. (a) The representative images observed at 0 h, 6 h, 12 h, and 24 h after the initial width of scratches of each group was about 2 mm. (b) The closure ratio analysis approach is used to calculate the healing rate: would closure (percent) = [(0 h scratch area − scratch area of different time point)/0 h scratch area] × 100. A two-way ANOVA is used to analyze the data that come from three independent tests (scale bar = 2 mm).

**Figure 6:** Effects of P(VDF-TrFE) membranes with differential surface potentials on tube formation. (a) The representative images showed the effect of P(VDF-TrFE) membranes with differential surface potentials on the angiogenic ability of HUVECs. (b) Relative tube formation and master segments length were quantified by ImageJ software. A one-way ANOVA is used to analyze the data that come from three independent tests (scale bar = 200 *μ*m). ^∗^*p* < 0.05, ^∗∗^*p* < 0.01, ^∗∗∗^*p* < 0.001, and ^∗∗∗∗^*p* < 0.0001.

**Figure 7:** Effects of P(VDF-TrFE) membranes with differential surface potentials on gene expression. The results of VEGF-A and CD31 expression in HUVECs co-cultured with differential P(VDF-TrFE) membranes are summarized in this figure. The data from three independent tests were analyzed with a one-way ANOVA. ^∗^*p* < 0.05, ^∗∗^*p* < 0.01, ^∗∗∗^*p* < 0.001, and ^∗∗∗∗^*p* < 0.0001.

**Figure 8:** Effects of P(VDF-TrFE) membranes with differential surface potentials protein expression. As angiogenesis factors, VEGF-A (a) and CD31(b) protein expression levels were examined. The data from three independent tests were analyzed with a one-way ANOVA. ^∗^*p* < 0.05, ^∗∗^*p* < 0.01, ^∗∗∗^*p* < 0.001, and ^∗∗∗∗^*p* < 0.0001.

**Table 1:** Real-time PCR Primer sequences.

Genes	Forward primer sequences(5′-3′)	Reverse primer sequences(5′-3′)
GAPDH	GGAGTCCACTGGCGTCTTCA	GTCATGAGTCCTTCCACGATACC
VEGF-A	AGGGCAGAATCATCACGAAGT	AGGGTCTCGATTGGATGGCA
CD31	GGGAAGATGGTCGTGATCCTT	TCTGGGGTGGTCTCGATTTTA

## Data Availability

The data used to support the findings of this study are available from the corresponding author upon reasonable request.

## References

[1] Ducommun J., ElKholy K., Rahman L., Schimmel M., Chappuis V., Buser D. (2019). Analysis of trends in implant therapy at a surgical specialty clinic: patient pool, indications, surgical procedures, and rate of early failures-A 15-year retrospective analysis. *Clinical Oral Implants Research*.

[2] Aprile P., Letourneur D., Simonyarza T. (2020). Membranes for guided bone regeneration: a road from bench to bedside. *Advanced Healthcare Materials*.

[3] Kim O., Choi J., Kim B., Seo D. (2020). Long-term success rates of implants with guided bone regeneration or bone grafting. *Clinical Oral Implants Research*.

[4] Diomede F., Marconi G. D., Fonticoli L. (2020). Functional relationship between osteogenesis and angiogenesis in tissue regeneration. *International Journal of Molecular Sciences*.

[5] Chim S. M., Tickner J., Chow S. T. (2013). Angiogenic factors in bone local environment. *Cytokine & Growth Factor Reviews*.

[6] Hankenson K. D., Dishowitz M., Gray C., Schenker M. (2011). Angiogenesis in bone regeneration. *Injury*.

[7] Chen C., Bai X., Ding Y., Lee I.-S. (2019). Electrical stimulation as a novel tool for regulating cell behavior in tissue engineering. *Biomater. Res.*.

[8] Ryan C. N. M., Doulgkeroglou M. N., Zeugolis D. I. (2021). Electric field stimulation for tissue engineering applications. *BMC Biomed. Eng.*.

[9] Liu Z., Wan X., Wang Z. L., Li L. (2021). Electroactive biomaterials and systems for cell fate determination and tissue regeneration: design and applications. *Advanced Materials*.

[10] Tai G., Tai M., Zhao M. (2018). Electrically stimulated cell migration and its contribution to wound healing. *Burns & Trauma*.

[11] Zhao M. (2006). Electrical stimulation and angiogenesis. *The Cell Cycle in the Central Nervous System*.

[12] Bai H., Forrester J. V., Zhao M. (2011). DC electric stimulation upregulates angiogenic factors in endothelial cells through activation of VEGF receptors. *Cytokine*.

[13] Li Y., Li X., Zhao R. (2017). Enhanced adhesion and proliferation of human umbilical vein endothelial cells on conductive PANI-PCL fiber scaffold by electrical stimulation. *Materials Science and Engineering: C*.

[14] Liu W., Li X., Jiao Y. (2020). Biological effects of a three-dimensionally printed Ti6Al4V scaffold coated with piezoelectric BaTiO_3_ nanoparticles on bone formation. *ACS Applied Materials & Interfaces*.

[15] Gan W. C., Abd Majid W. H., Furukawa T. (2016). Ferroelectric polarization, pyroelectric activity and dielectric relaxation in form IV poly(vinylidene fluoride). *Polymer*.

[16] Hitscherich P., Wu S., Gordan R., Xie L. H., Arinzeh T., Lee E. J. (2016). The effect of P(VDF-TrFE) scaffolds on stem cell derived cardiovascular cells. *Biotechnology and Bioengineering*.

[17] Bai Y., Dai X., Yin Y. (2019). Biomimetic piezoelectric nanocomposite membranes synergistically enhance osteogenesis of deproteinized bovine bone grafts. *International Journal of Nanomedicine*.

[18] Augustine R., Dan P., Sosnik A. (2017). Electrospun poly (vinylidene fluoride-trifluoroethylene)/zinc oxide nanocomposite tissue engineering scaffolds with enhanced cell adhesion and blood vessel formation. *Nano Research*.

[19] Damaraju S. M., Shen Y., Elele E. (2017). Three-dimensional piezoelectric fibrous scaffolds selectively promote mesenchymal stem cell differentiation. *Biomaterials*.

[20] Metwally S., Stachewicz U. (2019). Surface potential and charges impact on cell responses on biomaterials interfaces for medical applications. *Materials Science and Engineering: C*.

[21] Burke M., Armstrong J. P. K., Goodwin A. (2017). Regulation of scaffold cell adhesion using artificial membrane binding proteins. *Macromolecular Bioscience*.

[22] Chang H.-Y., Huang C.-C., Lin K.-Y. (2014). Effect of surface potential on NIH3T3 cell adhesion and proliferation. *The Journal of Physical Chemistry C*.

[23] Metwally S., Ferraris S., Spriano S. (2020). Surface potential and roughness controlled cell adhesion and collagen formation in electrospun PCL fibers for bone regeneration. *Materials & Design*.

[24] Zhao W., Cui W., Shujun X., Cheong L.-Z., Wang D., Shen C. (2019). Direct study of the electrical properties of PC12 cells and hippocampal neurons by EFM and KPFM. *Nanoscale Advances*.

[25] Chang H.-Y., Kao W.-L., You Y.-W. (2016). Effect of surface potential on epithelial cell adhesion, proliferation and morphology. *Colloids and Surfaces B: Biointerfaces*.

[26] Zhu P., Lai C., Cheng M. (2022). Differently charged P(VDF-TrFE) membranes influence osteogenesis through differential immunomodulatory function of macrophages. *Front Mater*.

[27] Ahn H. H., Lee I. W., Lee H. B., Kim M. S. (2014). Cellular behavior of human adipose-derived stem cells on wettable gradient polyethylene surfaces. *International Journal of Molecular Sciences*.

[28] Amani H., Arzaghi H., Bayandori M. (2019). Controlling cell behavior through the design of biomaterial surfaces: a focus on surface modification techniques. *Advanced Materials Interfaces*.

[29] Lee Y.-S., Arinzeh T. L. (2012). The influence of piezoelectric scaffolds on neural differentiation of human neural stem/progenitor cells. *Tissue Engineering Part A*.

[30] Szewczyk P. K., Metwally S., Karbowniczek J. E. (2019). Surface-potential-controlled cell proliferation and collagen mineralization on electrospun polyvinylidene fluoride (PVDF) fiber scaffolds for bone regeneration. *ACS Biomaterials Science & Engineering*.

[31] Michaelis U. R. (2014). Mechanisms of endothelial cell migration. *Cellular and Molecular Life Sciences*.

[32] Carmeliet P., De Smet F., Loges S., Mazzone M. (2009). Branching morphogenesis and antiangiogenesis candidates: tip cells lead the way. *Nature Reviews. Clinical Oncology*.

[33] Zhao M., Bai H., Wang E., Forrester J. V., McCaig C. D. (2004). Electrical stimulation directly induces pre-angiogenic responses in vascular endothelial cells by signaling through VEGF receptors. *Journal of Cell Science*.

[34] Monteiro H. P., Maria T. O., Albuquerque M., Rocha Oliveira C. J., Curcio M. F., Luz P. L., Libby P., Chagas A. C. P., Laurindo F. R. M. (2018). Chapter 3 - signal transduction pathways in endothelial cells: implications for angiogenesis. *Endothelium and Cardiovascular Diseases*.

[35] Karaman S., Leppänen V.-M., Alitalo K. (2018). Vascular Endothelial Growth Factor Signaling in Development and Disease. *Development*.

[36] Zhao X., Guan J.-L. (2011). Focal adhesion kinase and its signaling pathways in cell migration and angiogenesis. *Advanced Drug Delivery Reviews*.

[37] Zhao Q., Lu W. W., Wang M. (2017). Modulating the release of vascular endothelial growth factor by negative-voltage emulsion electrospinning for improved vascular regeneration. *Materials Letters*.

[38] Marchesano V., Gennari O., Mecozzi L., Grilli S., Ferraro P. (2015). Effects of lithium niobate polarization on cell adhesion and morphology. *ACS Applied Materials & Interfaces*.

[39] Chen W., Yu Z., Pang J., Yu P., Tan G., Ning C. (2017). Fabrication of biocompatible potassium sodium niobate piezoelectric ceramic as an electroactive implant. *Materials (Basel)*.

[40] Dubey A. K., Basu B. (2014). Pulsed electrical stimulation and surface charge induced cell growth on multistage spark plasma sintered hydroxyapatite-barium titanate piezobiocomposite. *Journal of the American Ceramic Society*.

[41] Xue G., Zhang Y., Xie T. (2021). Cell adhesion-mediated piezoelectric self-stimulation on polydopamine-modified poly(vinylidene fluoride) membranes. *ACS Applied Materials & Interfaces*.

[42] Moccia F., Negri S., Shekha M., Faris P., Guerra G. (2019). Endothelial Ca2+ signaling, angiogenesis and vasculogenesis: just what it takes to make a blood vessel. *International Journal of Molecular Sciences*.

